# A Research on the Establishment of a System Improving Teaching Ability of English Teachers in the Classroom Setting by Utilizing Artificial Intelligence

**DOI:** 10.1155/2022/8371437

**Published:** 2022-06-30

**Authors:** Xiaona Zhang

**Affiliations:** Jiyuan Vocational and Technical College, Jiyuan 459000, China

## Abstract

The efficient implementation of the artificial intelligence approaches could nobly resolve the deficiencies of the conventional approaches. This manuscript puts forward a scheme to construct a system that helps provide feedback on the teaching performance of English teachers in a classroom setting by utilizing artificial intelligence. Thus, the artificial intelligence-based framework is combined with the traditional system theories dealing with the teaching performance of English teachers in a classroom setting. For this purpose, the BP neural network is utilized to compute the teaching performance, which can effectively improve the teaching style in the classroom setting by updating the implemented teaching methodology, avoiding examination-oriented assessment, and increasing the multiorientation. To assure the rationality and effectiveness of the constructed scheme for English teachers, a simulation experiment is conducted. So, the teaching evaluation system of the English teachers is analyzed based on the constructed scheme. The experiment suggests that traditional system theories when combined with artificial intelligence schemes under the proposed scheme are found to be more suitable for modern English teaching activities in the classroom setting.

## 1. Introduction

Computerization has changed the way many disciplines are used to be implemented. Since continuous improvement and progression have taken place in the field of computers and their implementations, its functionality has gained momentum in various fields to present several favorable implementations. For example, one of them called artificial intelligence (AI), a novel way of crunching data, has been gaining momentum covering several subjects. Especially, the application of computers in the education discipline began in the 1980s. Even though the system theory dealing with the traditional teaching performance of English teachers in the classroom setting has achieved fruitful results, it is a fact that technological advancements could have the potential to bring more opportunities and improvements to the conventionally well-implemented methods, for example, the traditional system theory. So, the computer-aided (CAI) systems help attain better results for the performance of English teaching in the classroom setting; for example, the contemporary fast multidimensional teaching mode is one of them when the current technology and science level is under consideration [1], which requires to develop an assessment changing from a single dimension to multidimensional one with an effective change [1]. On the other hand, this change could bring pressure on English teachers. Even though the multiangle approach gets started to enhance the quality of classroom teaching, thus, improving the ability of students to have more sensory acceptance [2], they have several difficulties associated with it. When compared with computer-aided teaching, artificial intelligence system in classroom teaching provides certain reasoning abilities.

The BP neural network, one of the AI methods, introduced in artificial intelligence has wide application areas and contributes to the development of better approaches and research directions in several disciplines. So, this manuscript will utilize it to propose a construction scheme for English teachers to improve classroom teaching [3].

AI systems are utilized for better teaching in the classroom and better representation of knowledge systems, providing expert teaching systems and virtual reality and eventually an improved learning environment and intelligent help system when the classroom education is a concern [2]. Significant improvements have been achieved when intelligent systems and their implementation in classroom teaching are concurrently implemented. Especially, it could be utilized to both improve the quality of classroom teaching and promote the multisensory acceptance abilities of students [4]. The findings suggest that the impact could be remarkable in some respects. Nevertheless, several issues were found to be dealt with when more research was conducted. For instance, contemporary artificial intelligent systems are mostly characterized by expressions such as simple and difficulty expressing their contents, not being an easy formalization of procedural knowledge. Besides, students' roles are defined generally as passive recipients of knowledge when an ordinary classroom setting is under consideration. Thus, students lack interaction. On the other hand, optimizations of such a system are needed. Thus, more comprehensive research is required.

This manuscript presents the AI technology and applies it to the classroom setting to improve teaching. For this purpose, the BP neural network is utilized to compute the performance of the teaching activities in classrooms, which could efficiently enhance it when changes occur in teaching methodologies, avoid the classroom teaching mode of examination-oriented assessment, and increase the multidirectional teaching.

## 2. Preliminary to Artificial Intelligence

### 2.1. Fundamentals of Artificial Intelligence

The implementation of AI to establish a system that feeds back on the teaching performance of English teachers is one of the research areas where the AI contributes much and reforms English teaching. To conduct this type of implementation, data is the main source and is collected by computers utilizing sensors or manual input. Then, the collected data is stored and updated and finally compared to extract insights. Then, computations are finally conducted to determine diverse possible options to utilize and predict which one is relatively the best one. AI process can be defined from a human being's point of view as follows: the surroundings of human beings play stimulation roles, and responses correspondingly occur. Thus, learning, inferences, judgments, and other mental processes are realized. Therefore, some simple basic procedures are generated by gradually running the decomposition of these processes. Finally, the constructed intelligent design and the responses to outside stimulations generated by human beings are concurrently employed to resolve the real problems that human beings face.

An intelligent system is a structured method that mimics the processes used by human beings to devise and resolve complicated issues systematically. Thus, a set of software-based tools takes the place of the processes utilized by human beings to resolve the given problems. The simplified form of the schema is depicted in Figure 1.

Figure 1 is just a generic representation of the AI system that mimics the processes employed by human beings to realize the learning process. This manuscript proposes an AI system consisting of several parallel and independent sensors. Different design structures can be employed to increase the capacity of the system too. Then, the related computing power would be increased. The components of an AI system consist of a memory, a logic operator, an operation editor, a logic module power supply, and a control separation system [2].

Besides, to attain fast logical operations, the selection of the carrier position needs the operation rate with the largest value [2].  Figure 2 depicts it below.

Figure 2 suggests that when the carrier position is between 8 and 10, the calculation speed tends to be the largest, and then, the reconstructed AI could be introduced into the capacity system of English teaching.

### 2.2. Introduction of AI

The conventional teaching setting needs to be redesigned when a relatively complicated AI-based process is under consideration. Computer-based intelligence is expected to help and increase the performance of human intelligence in a better way to attain more refined outcomes, which is called an auxiliary tool. Thus, the contribution of the AI systems formalizes the process of knowledge better. Besides, AI could also be employed for other purposes such as retrieving knowledge, conducting reasoning, and making inferences; namely, knowledge processing with automation and intelligence is realized.

Hence, AI could have a crucial role in redesigning the classroom teaching of English teachers to obtain better performances [5]. When the implementation of an AI system used for feedbacking to English teachers is under consideration, the different situations and different aptitudes of each student should be considered to fit [5]. The modules of “teaching decision,” the “student model,” and the “natural language interface” are called the components of this system [2]. For after-school counseling, test simulation, and daily practice, sessions covering various teaching modes are utilized to give a full play to conduct activities whose characteristics should be interactive and self-phased methods [2]. When AI is implemented in a teaching system that provides feedback on the classroom teaching performance of English teachers, Figure 3 depicts it in detail below.

Figure 3 depicts the flowchart of the AI-based system implemented in classroom teaching. Data is acquired first. If it can be readily usable, then it is sent to the teaching data interface, otherwise, a preprocessing step is conducted. Afterward, data analysis is run based on an AI-based approach. Then, the data processor steps deal with data analysis back and forth to make it ready for display. Finally, the database system is updated based on the current outcomes.

AI system could be more useful when the data analysis module is integrated. The data analysis module helps increase the performance of artificially intelligent systems. First of all, we compute weights that will be used in the next phase of the proposed model. Equation (1) presents it.

(1) $$\begin{array}{c} W_{i}=\frac{\left[R‐b_{i}^{-p}/R\text{c}\right]}{\sum_{i=1}^{n}{\left[R‐a_{i}^{-p}/R\text{c}\right]}_{i}^{2}}. \end{array}$$

The weight, *W*_i_, is computed to denote the momentum of intelligence [2]. *R* denotes the volume of the database; *b*_*i*_^−*p*^ represents the execution variable of AI, *R*c represents the energy variables of the database; *a*_*i*_^−*p*^ denotes the expression variable of the artificial attribute. Thus, *i*th weight can be computed for the system.

When weights are computed by crunching the database [6], the first phase of constructing the AI system is finalized. The weights will be used in the next set of equations.

## 3. Using Artificial Intelligence to Rebuild Classroom Teaching of English Teachers

The software design also needs to be optimized for the two major software systems. While the first is called the teaching management system, the second is called the teaching system. These two systems need to achieve real-time data collection, analysis, and processing. Besides, they need two systems to complement each other to ensure the integrity of teaching while achieving personalized teaching configuration. BP neural network is introduced to optimize data processing.

### 3.1. Introduction of BP Neural Network

To assure an orderly teaching process,

(2) $$\begin{array}{c} Y_{j}=\frac{1}{1+\exp\left[‐\left(\sum_{i=1}^{n}\omega_{ij}x_{i}-\theta_{j}\right)\right]}, \end{array}$$

where *i* = 1, 2, ⋯, *n* and *j* = 1, 2, ⋯, *s* [7].

*Y*_j_ refers to the valid weight parameter of the overall data identification for the knowledge data end, which can be parameterized so that it can guarantee the control capability; *ω*_*ij*_ is called weighted connection weights; *x*_*i*_ refers to the input value of the iteration input layer; *θ*_*j*_ refers to input layer's feedback level threshold.

The significance of data processing in the data port related to teaching is aimed at obtaining a higher evaluation of teaching quality. By analyzing the influence of various factors that have an impact on the teaching quality, the final summary data is obtained and the data are processed and correctly divided into grades. Thus, the following indicators are obtained from the overall teaching point of view as follows:

(3) $$\begin{array}{c} \text{Teaching attitude}\left\{\begin{array}{c} \text{Complete lesson preparation}\\ \text{Counseling Q}\&\text{A and correcting homework} \end{array}\right.\\ \text{Teaching attitude}\left\{\begin{array}{c} \text{Rationality of selection of teaching materials}\\ \text{Scientific and accurate}\\ \text{Outstanding key and difficult points} \end{array}\right.\\ \text{Teaching attitude}\left\{\begin{array}{c} \text{Specified language},\text{clear interpretation and suitable blackboard}\\ \begin{array}{c} \text{Use advanced and scientific teaching meansTeach according to }\\ {\text{students}}^{\text{'}}\text{ aptitude and enlightening} \end{array} \end{array}\right.\\ \text{Teaching effect}\left\{\begin{array}{c} \text{Mastery of knowledge}\\ \text{Cultivation of ability} \end{array}\right. \end{array}$$

The evaluation system to measure the quality of teaching is established employing those indexes, which provide a methodological basis for the establishment of the BP neural network model [8]. Then, these constructs are utilized to establish the BP neural network model that will be employed to construct a system to evaluate English teachers' performance in a classroom teaching system, which is mainly related to the efficiency of learning [9]. The structure of the BP neural network can be defined by [10]. Equation (4) represents the four-layered BP neural network.

(4) $$\begin{array}{c} T_{S_{\text{tuck}}}\left(\text{R},\text{T}\right)=\left\{\begin{array}{c} \exp\left(\frac{‐{\left(\beta_{y}‐\eta_{y}/2‐R-y\right)}^{2}}{\left(2S_{y}^{2}\right)}\right)\;\text{if}\left(x,y\right)\in H_{\text{ETR}1},\\ \exp\left(\frac{‐{\left(\beta_{x}‐\eta_{y}/2‐R-x\right)}^{2}}{2S_{y}^{2}}\right)\;\text{if}\left(x,y\right)\in H_{\text{ERT}2},\\ \exp\left(\frac{‐{\left(\beta_{y}+\eta_{y}/2+R-y\right)}^{2}}{\left(2S_{y}^{2}\right)}\right)\;\text{if}\left(x,y\right)\in H_{\text{ERT}3},\\ \exp\left(\frac{‐{\left(\beta_{x}+\eta_{y}/2+R-x\right)}^{2}}{\left(2S_{y}^{2}\right)}\right)\text{if}\left(x,y\right)\in H_{\text{ETR}4}, \end{array}\right. \end{array}$$

where *H*_ETR1_, *H*_ERT2_, *H*_ERT3_, and *H*_ETR4_ stand for the four levels of the network for the learning phase; this level is divided according to the total times of training within the different periods and can be adjusted manually; *x* and *y* stand for the horizontal and vertical coordinate values of the BP neural network to calculate the model; *β* refers to the connection weights of the vertical and horizontal coordinates related to input layers; *η* stands for the neuronal thresholds for implicit layers of horizontal and vertical coordinates.

Afterward, data processing should be conducted as follows:

(5) $$\begin{array}{c} \frac{\partial^{2}N_{2}}{\partial i^{2}}=\frac{\left(L-L_{\text{m}}‐N_{2}\right)W_{0}\left(i\right)}{w_{0}\left(i\right)}≻0,\\ \frac{\delta L_{\text{m}}}{\delta i}=\frac{\left(L-L_{\text{m}}‐N_{2}\right)W_{0}\left(i\right)\left(L‐N_{i}\right)}{A+w_{0}\left(i\right)\pi }≻0, \end{array}$$

where *∂*^2^*N*_2_ refers to the trend of the data collected by the artificial intelligence system; *∂i*^2^ characterizes the processed artificial intelligence predictive constant; *W*_0_ denotes the big data collection analysis; *L*_m_ refers to the data simulation model index; and *A* refers to planning data coefficients.

After running the steps, the hardware and software processing and optimization of the BP neural network were conducted. Finally, the processed data needs to be classified and managed. The process is expressed as follows:

(6) $$\begin{array}{c} \frac{\min{\left\{E_{C}^{2}\left[{\overset{⌢}{P}}_{\text{OBYT}-1},{\overset{⌢}{P}}_{\text{OBYK}}\right]\right\}}_{T=R}^{S}}{2\sigma }=\frac{\underset{R}{\min}{\left\{E_{\text{i}}^{2}\left[{\overset{⌢}{P}}_{\text{OBYK}-1},\overset{T}{{\overset{⌢}{P}}_{\text{OBYK}}}\right]\right\}}_{i=R}^{S}}{2\sigma }=\frac{\underset{S}{\min}{\left\{F_{S}^{2}\left[{\overset{⌢}{P}}_{\text{OBYT}-1},\overset{S}{{\overset{⌢}{P}}_{\text{OBYT}}}\right]\right\}}_{i=T}^{T_{\text{i}}}}{2\sigma }=‐\ln\Delta \alpha_{\text{MAX}}, \end{array}$$

where *E*_*C*_^2^ refers to conditions to process and run the data, which can comprehensively classify the data; 2*σ* denotes the usage reference parameter of the networking momentum; ${\overset{⌢}{P}}_{\text{OBYT}-1}$ presents the initial step pace of the moment, which can effectively classify the judgment data; ${\overset{⌢}{P}}_{\text{OBYK}}$ refers to the total iteration times of the data; and *E*_*i*_^2^ denotes the conditions to use high-order data classification. The data are separated by this condition; *F*_S_^2^ represents the effective expression of data classification [3]. The calculation process regarding the BP neural network is depicted in Figure 4.

### 3.2. The Reconstruction of the Teaching Ability System

Devising a system that feeds back on the classroom teaching performance of English teachers in this paper is mainly aimed at measuring oral expression ability and listening comprehension. Therefore, the voice recognition ability determines the utilization of the system. For its use, the validity of the audio data is conducted, and the process is defined as follows:

(7) $$\begin{array}{c} \omega_{j}\left(t+1\right)=\omega_{j}\left(t\right)+\eta \left(t\right){oy}_{j}+\alpha \left[\omega_{j}\left(t\right)-\omega_{j}\left(t-1\right)\right],\\ \theta \left(t+1\right)=\theta \left(t\right)+\eta \left(t\right)\sigma +\alpha \left[\theta \left(t\right)-\theta \left(t-1\right)\right],\\ n_{\left(t\right)}=\eta \left(0\right)\left[1-\frac{t}{T+M}\right], \end{array}$$

where *ω*_*j*_(*t* + 1) refers to the effective recognition of voice data, which can be used to measure the standard data related to speech; *η*(*t*) denotes effective recognition of audios whose parameter needs adjustment to some extent; *y*_*j*_ refers to the storage of the voice database used for English teaching; *T* refers to the conversion coefficient; *o* represents the storage quantity; and *M* refers to the coefficient of a connection weight.

If the data recognition requirements for data storage can be met, the evaluation level of the input lever factors can be modified and balanced to compute the assessment system of the proposed method represented by

(8) Sx=ATS−1A−1=R11⋯ R1n        Rn1 ⋯Rnn, n=1,2,⋯,N−2.

*S*_*x*_ denotes the upper limit of the real correction bias of the data obtained by the teaching system; *A*^*T*^ refers to the expected output data of the deviation; *S*^−1^ represents the error quality parameter. After conducting modification, all data can be employed to construct the proposed system. Equation (9) presents the process defined by

(9) $$\begin{array}{c} F\left(E_{T}\left|A_{R}^{\left(i\right)},b\right.\right)\infty \exp\left(\frac{‐F_{T}^{2}\left[{\overset{⌢}{P}}_{\text{OBY},S-1},\overset{i}{{\overset{⌢}{P}}_{\text{OBY},S}}\right]}{2\beta }\right), \end{array}$$

(10) $$\begin{array}{c} E\left(b\right)\infty P_{f}^{2}\left[{\overset{⌢}{P}}_{\text{OBY},S-1},\overset{i}{{\overset{⌢}{P}}_{\text{OBY},S‐1}}\right]=\frac{E_{f}^{2}\left[{\overset{⌢}{P}}_{\text{OBY},S-1},\overset{i}{{\overset{⌢}{P}}_{\text{OBY},S}}\right]}{\sum_{f\in \left\{S,R,T\right\}}F_{f}^{2}\left[{\overset{⌢}{P}}_{\text{OBY},S-1},\overset{i}{{\overset{⌢}{P}}_{\text{OBY},S}}\right]}. \end{array}$$

*E*_*T*_ refers to the effective matrix condition reconstructed by data, which can be stored at the cloud end of the knowledge network database; *A*_*R*_^(*i*)^ represents the momentum reference coefficient calculated by the BP neural network; *F*_*T*_^2^ denotes a collection of feature sets; 2*β* presents the initial pace length; and *P*_*f*_^2^ refers to the data partition of the distribution of information texture set [5].

## 4. Simulation

To assure the validity of the constructed scheme, a comparative simulation experiment is designed [11]. Besides, to ensure the validity of the experiment, the conventional system used by English teachers in the classroom setting is employed by combining with artificial intelligence.

### 4.1. Parameter Setting

The parameters are set as follows: the implemented weight parameters *Y*_*j*_ for the overall data recognition to the knowledge data end are assigned to [35.8-54.7]; *H*_ETR1_, *H*_ERT2_, *H*_ERT3_, and *H*_ETR4_ are set to 1000, 2000, 3000, and 4000, respectively.

This experiment contains several random and sudden factors. Random and sudden factors mean that they abruptly occur when the simulation is run due to causes that were not considered or their measurements cannot be added significantly to the system. Therefore, there exist certain inherent changes randomly occurring in the teaching environment, which are depicted in Figure 5.

### 4.2. The Correction of Data Error in the Experiment

Another phase that needs to be run is to optimize and adjust the data concerning some uncertain factors occurring in the experiment process.  Table 1 summarizes and refers to the General Qualification Data Sheet.

### 4.3. The Results of the Experiment

Two methods were employed to record the comprehensive scores of randomly conducted simulation for English teaching, whose outcomes are presented in Table 2.

After error adjustment is conducted, a line chart is obtained and presented as follows.

Figure 6 depicts that the constructed scheme provides better outcomes in the classroom teaching of English teachers utilizing AI when compared with the conventional one [2].

When the criteria such as the evaluation of English teaching and teaching completeness are a concern, the three-dimensional coordinate system represents the outcomes better as follows.

Figure 7 depicts the system that feeds back the classroom teaching scores of English teachers utilizing the AI-based method in this manuscript [5]. By doing so, the proposed method could transform the conventional system with a single dimension into a multidimension effectively and could, however, bring a quite amount of stress to English teachers. Nevertheless, the implemented multidimensions system could enhance the teaching quality in the classroom.

In consequence, this manuscript devises a scheme that provides feedback to English teachers to perform better teaching quality by converting the ordinary system with a single dimension to a multidimension effectively. Besides, this multiangle scheme could promote students' multisensory acceptance. Thus, it is found to be more favorable to utilize when teaching English in the classroom setting [5].

## 5. Conclusion

A system combined with AI providing feedback on the classroom teaching performance of English teachers is proposed in this manuscript. This system extends a single dimension assessment scheme to multidimensions that eventually make the classroom teaching performance of English teachers reach a more effective level. Thus, a high level of liberation could be brought to English teachers, and the teaching quality could be improved. Besides, students' multisensory acceptance could be promoted.

One of the AI methods, the BP neural network, is utilized to compute the assessment of classroom teaching, which could effectively improve the classroom teaching performance when the teaching method of examination-oriented approach is avoided. To ensure the rationality and effectiveness of the proposed method, a simulation experiment is conducted that found that the proposed system contributes more efficiency to the contemporary classroom teaching of English.

## Figures and Tables

**Figure 1:** The simplified chart of artificial intelligence design.

**Figure 2:** Relationship between carrier position and operation rate.

**Figure 3:** Artificial intelligence chart in the classroom teaching.

**Figure 4:** The calculation process of the BP neural network.

**Figure 5:** The frequency chart showing inherent fluctuations regarding teaching.

**Figure 6:** The comparison of the results.

**Figure 7:** The results of the comprehensive evaluation of the proposed methods.

**Table 1:** Data for reference.

	Adjustment limit/*N*	Storage limit/*J*
1	26.8	19.5
2	27.9	20.3
3	29.3	20.5
4	28.9	19.0
5	29.0	19.6
6	30.3	19.8

**Table 2:** The experimental results.

Times of experiment	The proposed method	Traditional method
1	7.8	5.5
2	7.4	5.4
3	8.2	4.9
4	8.5	5.2
5	8.2	5.9
6	8.0	6.0

## Data Availability

Data will be available upon request to the author.
